The article "Difference in leg asymmetry between female collegiate athletes and recreational athletes during drop vertical jump" was published in 2019. Journal: J Orthop Surg Res.

# Difference in leg asymmetry between female collegiate athletes and recreational athletes during drop vertical jump

**DOI:** 10.1186/s13018-019-1490-5

**Published:** 2019-12-10

**Authors:** Yutaro Morishige, Kengo Harato, Shu Kobayashi, Yasuo Niki, Morio Matsumoto, Masaya Nakamura, Takeo Nagura

**Affiliations:** 1 Department of Orthopedic Surgery, Keio University School of Medicine, Tokyo, Japan; 2 Department of Clinical Biomechanics, Keio University School of Medicine, 35 Shinanomachi, Shinjuku-ku, Tokyo, 160-8582 Japan

**Keywords:** Anterior cruciate ligament, Lower extremity, Non-contact injury, Exercise intensity, Asymmetric motion, Leg dominance, Jump task

## Abstract

**Background:**

Neuromuscular imbalance will lead to loading asymmetry in sporting activities. This asymmetry is related to leg dominance, which has been associated with increased risk of anterior cruciate ligament (ACL) injury. Therefore, potential biomechanical differences between legs are important. However, little attention has been paid to the biomechanical details of leg dominance. The purpose of the present study was to clarify the relationship between leg dominance and knee biomechanics in females with different activity level during dynamic athletic tasks.

**Methods:**

A total of 23 female collegiate (mean age = 19.6 ± 1.4 years, mean body mass index = 21.5 ± 0.9) and 19 recreational athletes (mean age = 20.7 ± 1.1 years, mean body mass index = 20.5 ± 1.7) were enrolled. Tegner activity scores of the collegiate and recreational athletes were 9 and 7, respectively. Knee kinematic and kinetic asymmetries between the dominant (DL) and non-dominant (NDL) legs during the landing phase of drop vertical jump (DVJ) were assessed using three-dimensional motion analysis in collegiate and recreational athletes separately. Statistical comparison was done using two-tailed paired *t* test between DL and NDL in each athlete.

**Results:**

The peak knee abduction angle was significantly larger on the DL than on the NDL in collegiate athletes. Knee abduction angle at initial contact (IC), peak knee abduction angle, knee internal rotation angle at IC, and peak knee internal rotation angle were significantly larger on the NDL than on the DL in recreational athletes. Moreover, peak knee abduction moment within 40 ms from IC was larger on the NDL than on the DL in recreational athletes, while the moment was not significantly different in collegiate athletes.

**Conclusions:**

From the present study, the relationship between leg dominance and knee biomechanics was totally different in females with different activity level. Specifically, asymmetry of the knee abduction angle between limbs was opposite between female recreational and collegiate athletes. According to previous literatures, abduction and internal rotation angles as well as abduction moment were key issues for mechanism of non-contact ACL injury. Therefore, the NDL in female recreational athletes was associated with increased risk of ACL injury.

## Background

Leg dominance in sports leads to loading asymmetry and can contribute to the development of unilateral damage to the lower limbs such as anterior cruciate ligament (ACL) injuries, especially in females [1–3]. About 70 to 80% of ACL tears involve non-contact injuries such as landing from a jump, a quick stop, or a cutting maneuver [4]. Moreover, female athletes were at greater risk of ACL injury than male athletes in non-contact sports [5]. According to previous studies, leg dominance is an important factor in non-contact ACL injuries [6–8]. For instance, Brophy et al. reported that 68% of females were injured on the non-dominant leg (NDL) and 74% of males were injured on the dominant leg (DL) in ACL injury during soccer [6]. In addition, Ruedl et al. reported that female recreational skiers suffered more often from non-contact ACL injuries on the NDL than male recreational skiers; however, there was no difference on the DL [8], although conclusions have remained inconsistent. Based on a previous study, physical performance including vertical jump might be reduced by inter-limb asymmetries [9]. For this reason, loading asymmetry has been associated with the intensity and frequency of sporting activities.

Drop vertical jump (DVJ) provides a useful screening test for the risk of non-contact ACL injuries in females [10]. The DVJ requires an athlete to drop from a static box, land, and immediately execute a maximal vertical jump. Based on kinematic and kinetic performance traits and anatomical variables, an algorithm has been designed using the DVJ to evaluate the cumulative risk of non-contact ACL injury [10]. The DVJ has thus been used as a method of evaluating the risk of ACL injury in various studies [11–22]. Although, the DVJ is a double-limb landing task, limb asymmetry, which is an established factor for repeated ACL injury, is evident during this test [2]. However, little is known about the effects of asymmetric knee kinematics and kinetics during DVJ in females who participate in sports at different level of intensity.

The purpose of the present study was to clarify the effects of leg dominance on the biomechanics of DVJ among healthy female collegiate and recreational athletes. It was hypothesized that loading condition would be different between female recreational athletes and collegiate athletes during DVJ.

## Methods

### Participants

All participants in the current study were recruited by personal contacts of the authors. The participants in the present study comprised 23 female collegiate athletes (mean age, 19.6 ± 1.4 years; height, 1.61 ± 0.05 m; weight, 56.3 ± 4.4 kg; basketball players, *n* = 15; soccer players, *n* = 8; mean competition history, 7.5 ± 4.3 years) and 19 female recreational athletes (mean age, 20.7 ± 1.1 years; height, 1.61 ± 0.06 m; weight, 53.2 ± 4.8 kg; basketball players *n* = 10; volleyball players, *n* = 9; mean competition history, 5.5 ± 3.7 years) (Table 1). Twenty-three female collegiate athletes were part of the Keio University Athletic Association, and 19 female recreational athletes were medical students of Keio University School of Medicine. Tegner activity scores among the collegiate and recreational athletes were 9 and 7, respectively. Based on practice schedule, we observed the actual practice and confirmed that physical demands in collegiate athletes were 3 h a day, five times a week, and those in recreational athletes were 3 h a day, three times a week, respectively. The dominant leg was the right side for all participants except for one participant in each group. As female athletes were at greater risk of ACL injury than male athletes in non-contact sports [1, 2], females were chosen in the current study. None of the participants had a history of major injury to the trunk or lower extremities. All of the athletes provided written informed consent to participate in this study, which was approved by our institutional review board (#20080054).

**Table 1:** Subject demographics (mean ± S.D.)

	Collegiate athletes (*n* = 23)	Recreational athletes (*n* = 19)	*P* value^a^
Age (years)	19.6 ± 1.4	20.7 ± 1.1	0.008
Height (m)	1.61 ± 0.05	1.61 ± 0.06	0.650
Weight (kg)	56.3 ± 4.4	53.2 ± 4.8	0.034
Body mass index (kg/m^2^)	21.5 ± 0.9	20.5 ± 1.7	0.022
Dominant leg (right/left)	22/1	18/1	
Tegner activity level scale	9	7	

^a^Values obtained using the two-tailed unpaired *t* test

### Test procedures

We defined DVJ as jumping from a 30-cm high box onto force plates positioned 50% of the height of each athlete away from the box and immediately rebounding on landing into a maximal vertical jump (Fig. 1). The participants were taught how to execute the DVJ and repeated the procedure several times before three trials were recorded. The DL was defined as the leg with which each athlete preferred to kick a ball [6–8]. We placed 46 retro-reflective markers (diameter, 14 mm) at standard anatomical landmarks in preparation for DVJ (Fig. 2). The following segments were tracked using three non-collinear infrared markers: two each for the feet, legs, and thighs, and one each for the pelvis and trunk. To define the axes of each of these eight segments, an anatomical model was created by digitizing the following standard bony landmarks: bilateral acromion processes, xiphoid process, suprasternal notch, 7th cervical vertebra, 10th thoracic vertebra, bilateral anterior and posterior superior iliac spines, bilateral iliac crests, bilateral greater trochanters, bilateral lateral and medial epicondyles, bilateral lateral and medial malleoli, bilateral posterior heels, bilateral medial cuneiforms, bilateral great toes, and bilateral heads of the 5th metatarsals. Four additional tracking markers were placed on each of the frontal aspects of the thigh and shank. Calibration markers (bilateral medial epicondyles and medial malleoli) were removed after the standing trial, and only tracking markers were left on the participants throughout all data collection.

**Fig. 1:** Setup of the laboratory for drop vertical jump. Drop landing task was defined as jumping from a 30-cm high box to a distance of 50% of their height away from the box onto force plates and immediately rebounding for a maximal vertical jump on landing

**Fig. 2:** Maker locations. A total of 46 retro-reflective markers (14 mm in diameter) were placed at standard anatomical landmarks

### Data processing and analysis

The DVJ was captured using a motion analysis system comprising eight Oqus cameras (Qualisys, Gothenburg, Sweden) at 120 frames/s and two AM6110 force plates with a frequency 600 Hz (Bertec, Columbus, OH, USA). The force plates collected data about ground reaction force (GRF) at 600 Hz and were synchronized to the camera sampling rate of 120 Hz. The time at initial contact (IC) and at toe-off (TO) from the jump were identified using the GRF. Three-dimensional kinematic, kinetic, and ground reaction force (GRF) data were recorded bilaterally during initial contact (IC) to toe-off (TO). Only data from the third trial were analyzed. The motions of markers were recorded using Track Manager version 2.7 software (Qualysis). We calculated knee kinematics and kinetics using Visual 3D (C-motion Co., Rockville, MD, USA). Knee flexion angle at IC, peak knee flexion angle, knee abduction angle at IC, peak knee abduction angle, knee internal rotation angle at IC, and peak knee internal rotation angle were adopted as kinematic parameters. Vertical ground reaction force (vGRF) (N), peak value of external knee flexion moment (PKFM) within 40 milliseconds (ms) from IC (Nm/kg), peak value of external knee abduction moment (PKABDM) within 40 ms from IC (Nm/kg), and peak value of external knee internal rotation moment (PKIRM) within 40 ms from IC (Nm/kg) were adopted as kinetic parameters. Furthermore, an increased risk of non-contact ACL injury was assessed for both limbs in each group. The definition of increased risk was positive value of knee abduction angle at IC and positive value of peak external knee abduction moment within 40 ms from IC based on previous studies [10–20]. The percentage of limbs with greater risk in each group was evaluated. Biomechanical asymmetry during both bilateral tasks was assessed as the absolute difference between the right and left leg for each data frame.

### Statistical analysis

Demographic data were compared between the female collegiate and recreational athletes using two-tailed unpaired *t* tests. Kinematic and kinetic data from DVJ were compared between the DL and the NDL within each group using two-tailed paired *t* tests. All data were statistically analyzed using SPSS® for Windows software (version 23; Microsoft, Chicago, IL, USA). Values of *P* < 0.05 were considered significant. A power analysis was performed using G*Power (v3.1.9.2, Heinrich-Heine University, Düsseldorf, Germany) in each group. Using a large effect size of 0.6 for one-way repeated measures of analysis of variance, a sample size of 19 was required in each group (*β* = 0.80, *α* = 0.05).

## Results

The collegiate athletes were significantly younger than the recreational athletes (*P* = 0.008) (Table 1). Similarly, the body mass index (BMI) was significantly larger in female collegiate than recreational athletes (*P* = 0.034).

In terms of kinematics, the knee flexion angle at IC was significantly smaller on the DL than on the NDL (*P* = 0.005) (Table 2), and peak abduction angle was significantly larger on the DL than on the NDL (*P* = 0.006) in collegiate athletes. The knee abduction angle at IC, peak knee abduction angle, knee internal rotation angle at IC, and peak knee internal rotation angle were significantly larger on the NDL than on the DL in female recreational athletes (*P* = 0.002, < 0.001, < 0.001, respectively).

**Table 2:** Kinematic and kinetic differences between DL and NDL (mean ± S.D.)

	Collegiate athletes		*P* value^b^	Recreational athletes		*P* value^c^
	DL	NDL		DL	NDL	
Knee flexion angle at IC (deg.)	33.0 ± 8.4	35.6 ± 8.3	0.005	35.5 ± 9.4	35.3 ± 11.2	0.868
Peak knee flexion angle at IC (deg.)	107 ± 12.9	109 ± 12.6	0.127	97.1 ± 12.6^d^	96.8 ± 13.0^d^	0.791
Knee abduction angle at IC (deg.)	− 2.1 ± 8.5	− 3.9 ± 6.8	0.143	− 4.8 ± 4.8	2.3 ± 4.9^e^	0.002
Peak knee abduction angle (deg.)	5.4 ± 11.8	1.5 ± 10.4	0.006	1.3 ± 7.2	6.3 ± 5.4	0.038
Knee internal rotation angle at IC (deg.)	− 7.6 ± 10.4	− 9.1 ± 9.1	0.400	− 12.4 ± 8.7	10.3 ± 8.2	< 0.001
Peak knee internal rotation angle (deg.)	4.4 ± 6.8	5.5 ± 6.7	0.557	0.0067 ± 7.0^d^	11.8 ± 5.4^e^	< 0.001
vGRF within 40 ms from IC (N)	1236 ± 629	1261 ± 366	0.827	1078 ± 314	1084 ± 445	0.953
PKFM within 40 ms from IC (Nm/kg)	1.69 ± 0.57	2.71 ± 0.88	< 0.001	1.67 ± 0.49	2.08 ± 0.87^d^	0.068
PKABDM within 40 ms from IC (Nm/kg)	0.36 ± 0.31	0.21 ± 0.36	0.827	0.17 ± 0.24^d^	0.38 ± 0.30	0.009
PKIRM within 40 ms from IC (Nm/kg)	0.16 ± 0.16	0.36 ± 0.39	0.675	0.22 ± 0.15	0.36 ± 0.39	0.175

^b^Values obtained using the two-tailed paired *t* test in collegiate athletes

^c^Values obtained using the two-tailed paired *t* test in recreational athletes

^d^Values were significantly larger in collegiate athletes than in recreational athletes using the two-tailed unpaired *t* test

^e^Values were significantly larger in recreational athletes than in collegiate athletes using the two-tailed unpaired *t* test

With respect to kinetic parameters, although vGRF did not significantly differ between limbs (*P* = 0.827), PKFM within 40 ms from IC was significantly smaller on the DL than on the NDL (*P* < 0.001) in collegiate athletes. Similarly, although vGRF did not significantly differ between limbs (*P* = 0.953), KABDM within 40 ms from IC was notably larger on the NDL than on the DL (*P* = 0.009) in the recreational athletes.

As to the differences between groups, peak knee flexion angle was significantly larger (*P* = 0.015), peak knee internal rotation angle was significantly larger (*P* = 0.047), and PKABM within 40 ms from IC was significantly larger in collegiate athletes, compared to recreational athletes on the DL. The peak knee flexion angle at IC was significantly larger (*P* = 0.0039), knee abduction angle at IC was significantly smaller (*P* = 0.0018), knee internal rotation angle at IC was significantly smaller (*P* < 0.001), peak knee internal rotation angle was significantly smaller (*P* = 0.0019), and PKFM within 40 ms from IC was significantly larger (*P* = 0.024) in collegiate athletes, compared to recreational athletes on the NDL.

Concerning the percentage of limbs that were at increased risk in each group, 10.5% on the DL and 73.7% on the NDL in female recreational athletes were at increased risk, while 30.4% on the DL and 21.7% on the NDL in female recreational athletes were at increased risk for non-contact ACL injury.

## Discussion

The present findings partly supported the hypothesis that loading condition would be different between female recreational athletes and collegiate athletes during DVJ. The most important finding in the present study was that the pattern of inter-limb kinematic asymmetry during DVJ was opposite between female collegiate and recreational athletes. Specifically, side-to-side asymmetry of the knee abduction angle during DVJ was opposite between female recreational and collegiate athletes.

According to the literature, valgus loading increases ACL force [23, 24] and leads to a key factor in the mechanisms of non-contact ACL injury. Hewett et al. reported that an increased knee abduction angle at IC, peak knee abduction angle, and peak knee abduction moment would correlate with increased risk for non-contact ACL injury during DVJ among female athletes [10]. In addition, rapid valgus and internal rotational development within 40 ms after IC is associated with ACL injury [25–27]. The present findings showed a greater internal rotation angle at IC, a greater peak knee internal rotation angle, and greater knee valgus loading on the NDL in female recreational athletes. As greater valgus loading and internal rotation angle were observed on the NDL, compared to the DL in female recreational athletes, the risk for non-contact ACL can be increased on the NDL in recreational athletes.

Neuromuscular asymmetry is related to primary and secondary non-contact ACL injury [1, 2, 10, 28–31]. For example, female athletes have higher side-to-side asymmetry for hamstring isokinetic torque and the ratio of hamstrings to quadriceps. Moreover, Pappas et al. found greater abduction angle and knee kinematic asymmetry in female than male athletes during forward landings [29]. Clinically, the incidence of non-contact ACL injury based on leg dominance has been reported. According to Brophy et al., 68% of females were injured on the NDL, while 74% of males were injured on the DL during soccer [6]. Moreover, Ruedl et al. suggested that female recreational skiers suffered more frequent from non-contact ACL injuries on the NDL than male recreational skiers, yet no difference was detected on the DL [8]. Therefore, the probability of injury on the NDL is higher among female than male recreational athletes. The present findings of female recreational athletes were thus similar to previous clinical studies in terms of increased risk of ACL injury on the NDL. According to a previous study, increased knee abduction angle and moment during DVJ were associated with an increased risk of non-contact ACL injuries [10]. Therefore, the NDL in female recreational athletes had the highest risk of non-contact ACL injury in this study (73.7%). On the other hand, the female collegiate athletes had greater risk of non-contact ACL injury on the DL, because the flexion moment was asymmetric and the peak knee abduction angle was larger on the DL than on the NDL. Sport-specific strategies to reduce asymmetry should be included in programs to prevent non-contact ACL injury.

Several limitations should be described in the current investigation. First, we could not match age and BMI between the groups. These differences might affect lower limb biomechanics. Second, although the risk of non-contact ACL injury was evaluated, the actual incidence of ACL injury could not be investigated. Third, the athletes participated in various sports, and thus, their background might have affected joint loading in the present study. In fact, Keio University School of Medicine does not have a female soccer team. Lastly, the true reason for biomechanical differences during DVJ between female collegiate and recreational athletes remains unknown, although collegiate athletes are more familiar with the jumping task methods that are commonly practiced among sports compared to recreational athletes. Nonetheless, the present results provide important information regarding the characteristics of female knee kinematics and kinetics with different activity level during jumping tasks.

## Conclusion

Asymmetry during DVJ differed between female collegiate and recreational athletes. Specifically, side-to-side asymmetry of the knee abduction angle and moment during DVJ were greater for female recreational athletes than female collegiate athletes. Therefore, the NDL in female recreational athletes is associated with increased risk of ACL injury. Hence, sport-specific asymmetry reduction should be incorporated into programs as a strategy to prevent injury during participation in recreational and collegiate sports.

## Data Availability

The datasets used and/or analyzed during the current study are available from the corresponding author on reasonable request.

## Abbreviations

ACL: Anterior cruciate ligament
DL: Dominant leg
DVJ: Drop vertical jump
GRF: Ground reaction force
IC: Initial contact
NDL: Non-dominant leg
PKABDM: Peak knee abduction moment
PKFM: Peak knee flexion moment
PKIRM: Peak knee internal rotation moment
TO: Toe-off
vGRF: Vertical ground reaction force
